RETRACTED

# Determinants of viral load suppression failure among HIV adults on ARV attending health care facilities: a retrospective study in Tanga region, Tanzania

**DOI:** 10.1186/s12879-023-08604-2

**Published:** 2024-03-14

**Authors:** Eric Mboggo, Expeditho Mtisi, Stella E. Mushy, Simon Mkawe, Frida Ngalesoni, Aisa Muya, Edwin Kilimba, Denice Kamugumya, Boniface Silvan Mlay

**Affiliations:** 1 AMREF Health Africa, Dar es Salaam, Tanzania; 2 Department of General Studies, Dar Es Salaam Institute of Technology, Dar es Salaam, Tanzania; 3 Department of Community Health Nursing, Muhimbili University of Health Science, Dar es Salaam, Tanzania; 4 Center for Disease Control and Prevention, Dar es salaam, Tanzania; 5 National AIDS Control Program, Ministry of Health, Dodoma, Tanzania

**Keywords:** Adult HIV positive, Antiretroviral therapy, DTG based therapy, HIV/AIDS, Viral load suppression, Predictors, Africa, Tanzania

## Abstract

**Background:**

Availability and accessibility of Antiretroviral drugs (ARV’s) improve the lives of People living with HIV (PLHIV) by improving client’s immune system to overcome infections and prevent the development of AIDS and other HIV complications. Combination therapy, early initiation of ART, newer ART drugs, single dosage and drug affordability significantly contribute in the reduction of viral multiplication and suppression of HIV to undetectable plasma levels.

**Methods:**

A retrospective longitudinal study design study was conducted from 1^st^ October, 2018 to 30^th^ June 2022 in all supported HIV care and treatment health facilities in Tanga region which were supported by Amref Health Africa, Tanzania. The participants were HIV adult patients aged 15 years and above on ART and attended the clinic at least once after ART initiation. Viral load suppression levels are defined with viral load <1,000 HIV RNA copies/ml (viral load suppression). Cox proportional hazard regression models were employed to identify risk factors for virological failure. *P* values were two-sided, and we considered a *P*<0.05 to be statistically significant.

**Results:**

Fifty-nine thousand five hundred three adult clients >15 years whom were on ART were included in the analysis to determine the level of plasma Viral Load suppression after being on ART. Female 41,304 (69.4%) and male 18,199 (30.6%). Only four percent (2,290) were found to be unsuppressed i.e having plasma Viral Load >1,000cp/ml while 96% (57,213) were virally suppressed. Several factors were independently associated with virologic failure that included; age between 15 - <25 years (HR: 2.82, 95% CI 1.96 – 4.04), BMI <18.5 (HR: 1.69, 95% CI 1.23 – 2.30), advanced WHO stage IV (HR: 1.60, 95% CI 1.12 – 2.24), CD4 cell count <350 (HR: 2.61, 95% CI 2.12 – 3.23), poor adherence (HR: 1.98, 95% CI 1.80 – 2.18) and not using DTG based drug (HR: 11.8, 95% CI 9.74 – 14.3).

RETRACTED

**Conclusion:**

Virologic failure was observed in this study among clients with young age, advanced WHO stage IV, not using DTG based regimen, poor drug adherence and second line regime. To improve Viral Load Suppression among these clients; the existing HIV intervention strategies should be taken care by targeting the identified risk factors.

## Introduction

Availability and accessibility of Antiretroviral drugs (ARV’s) improve the lives of People living with HIV (PLHIV) by improving client’s immune system to overcome infections and prevent the development of AIDS and other HIV complications [1]. Combination therapy, early initiation of ART, newer ART drugs, single dosage and drug affordability significantly contribute in the reduction of viral multiplication and suppression of HIV to undetectable plasma levels [1, 2].

Currently, 23.3 million people are on ART globally and those who started treatment earlier after being diagnosed have better progression as compared to those who started late with 43% reduction of mortality related to AIDS [3]. The effectiveness of HIV treatment is best monitored by measuring the amount of viral load in client plasma [3].

Tanzania Government has committed to mitigate the HIV/AIDS burden via introduction of National Stigma and Discrimination Strategy under Prime Minister’s Office as one of the road maps in curbing the epidemic [4]. The strategies aim to attain the three zero’s; zero new HIV infections, zero discrimination, and zero AIDS-related deaths. These can well be reached via mitigation of factors hindering HIV viral load suppression [3, 4].

Tanzania adapted the WHO criteria for viral load suppression levels where treatment success in HIV positive individuals is defined with viral load <1,000 HIV RNA copies/ml (viral load suppression) [5]. The low level of HIV Viral load help to reduce HIV related morbidity and mortality and improve the quality of life [4, 5]. According to UNAIDS fast track set goals of 95-95-95; the 3^rd^ 95 requires 95% of all clients on ART to be virally suppressed [6]. It’s estimated that, antiretroviral therapy coverage among people living with HIV in Tanzania has increase from 66% in 2018 to 86% in 2020 which is directly proportional to increase in viral suppression levels among PLHIV [7–9].

Viral load suppression is highly associated with reduced HIV morbidity and mortality and hence improve the lives of people living with HIV. Therefore, early detection of clients viral load status is key in attaining client’s clinical progression [10–12]. Virologic failure occurs earliest, followed by immunologic and lastly clinical failure. Timely detection of virologic levels with factors hindering viral suppression are essential in reducing the burden of HIV epidemic [1, 11–13].

RETRACTED

A study in sub-Saharan African country have demonstrated factors which are associated with virologic failure including age, gender, drug adherence, clinical appointment adherence, treatment interruption, ARV regimen, ART duration and occurrence of opportunistic infection especially Tuberculosis [1]. From the THIS 2017 report, 88% of adults aged 15 years and older on ART are Virally Suppressed where women (89.1%) outweigh male (84.4%). However, this achievement is far behind the global and national goal of 95% [3]. Meanwhile, UNAIDS 2022 recent report have shown 92% of people living with HIV have suppressed viral load in Tanzania [14].

This study aims to describe determinants associated with virologic failure among HIV adult patients on ART who are attending Care and Treatment Clinics in Tanga region, northern eastern part of Tanzania.

## Methodology

### Study design

A retrospective longitudinal cohort study of routine secondary HIV adult (>15 years old) data. Analytical secondary data were collected during routine visits including their viral load results at Care and Treatment Centers and were carried out using the electronic CTC2 database managed by the National Aids Control Program (NACP) [5].

### Study area and settings

The study involves all HIV/AIDS care and treatment sites in Tanga region, of Tanzania which are supported by Amref HIV care and treatment as implementing partners under Ministry of Health which are funded by Center for Disease Control and Prevention (CDC) from October, 2018 to June, 2022. As per the Tanzania HIV Impact Survey 2017, the HIV prevalence in Tanga is 5.0% (6.2% in women, 3.7% in men), among adults aging from 15 years and older. In such populations where HIV prevalence are such high, there may be increased prevalence and incidence of clinically detectable HIV secondary to virologic failure factors [3].

### Study population

The study population included all HIV adults (>15 years and older) whom were on ART at the time of the study attending routine CTC between 1^st^ October, 2018 to 30^th^ June, 2022. All the adults HIV clients were followed up during their usual CTC attendance. Their viral load results were collected and documented in the CTC2 database at their respective routine clinics.

Inclusion criteria considered all HIV adult clients (>15years) who were using ART at the time of the study and have their Viral load results returned and documented in the CTC2 database at their respective clinics.

RETRACTED

### Sample size and sampling technique

A total 59,503 HIV adult clients 15+ years and older on ART in Tanga region during the period of the study. All the records entered during their routine CTC clinic visits were used for analysis.

#### Variables

The dependent variable was Virologic failure rate. We collected information on adult age in years (15 - <25, 25 - <35, 35 - <45, 45 - <55 and 55+), Sex (male and female); Marital status (cohabitating, divorced, married and single), Districts (Handeni, Kilindi, Korogwe, Lushoto, Mkinga, Muheza, Pangani and Tanga); BMI (<18.5, 18.5 – <25, 25–<30 and 30+); WHO stage (I, II, III and IV); CD4 count cells/mm^3^ (<350, 350 - 500, 500+); ART duration in yrs (<=1, >1 yr); ART Adherence (good, poor); Virologic failure (No, Yes); Regimen (First line, Second line) and DTG based (Yes, No).

### Bias

The study was conducted using secondary data that have been collected in routine care and treatment visit clinic settings, which presented challenges in data quality, incompleteness and unmeasured confounders. To address these, data management and statistical techniques were engaged to review, identify and address data quality issues to minimize biasness.

### Statistical methods

Data were checked for completeness and consistency prior to analysis. The level of missing were assessed for each variable. Observations were excluded from analysis if data for the outcome variable were missing.

To determine the magnitude of Virologic failure in Tanga region, descriptive statistics were carried out and the frequencies and percentage of clients with HVL suppression level results were obtained. Proportion of client as per WHO staging, marital status, duration of ART usage and ART adherence were calculated to determine Virologic failure rate.

Cox proportional hazard model was employed to identify independent risk factors (sociodemographic and clinical characteristics) for Virologic failure. All significance tests were two-sided, and differences were considered significant at *p*-value less than or equal 0.05. Potential risk factors that were statistically significant at a *p*-value of 0.2 or less in univariate analysis were included as potential confounders in multivariate models. If the risk factor was binary, we used the Wald *p*-value from the regression output. If the risk factor was ordinal categorical, a single median score variable was created and use it in the model instead of multiple categories. If factor was nominal categorical variable, the Likelihood Ratio test was used. The missing indicator method was used to handle missing data. Statistical analysis was performed using the SAS ® statistical software package, Release 9.3 (Cary, North Carolina, USA).

RETRACTED

## Results

Figure 1, show flow of clients enrolled into the study from October 2018 to June 2022, a total of 61,651 HIV+ adult clients who were on ART at Tanga region were enrolled in a retrospective longitudinal study. Among these, 2,148 (3.5%) were excluded due to missing Viral load results, death and others being lost to follow up (LTFU). Ninety six point five percent, (59,503) adult clients >15 years whom were on ART were included in the analysis to determine the level of plasma Viral Load suppression after being on ART. Only four percent (2,290) were found to be unsuppressed i.e having plasma Viral Load >1,000cp/ml while 96% (57,213) were virally suppressed.

**Fig. 1:** Flow chart of CTC2 data for adults from 1^st^ October 2018 to 30^th^ June 2022 in Tanga

Table 1 shows the characteristics of the study population (*N*=59,503) of adult clients whom the median age group for participants was 44.2 (interquartile range, IQR: 36.1 – 53.2 years). Sixty nine point four percent were female while the rest 30.6% were male. Most clients (29%) came from Tanga Council followed by Muheza (19.3%) and Korogwe (16.4%) while the rest were from other councils across all Tanga region. According to facility level, we found that; most participants came from health centers (59.4%) followed by dispensary (22.4%) and hospital level (18.2%). Seventy six percent of clients had normal BMI (kg/m^2^) between 18.5 - <25 with only 4.5% being underweight <18, 12% having BMi between 25 - <30 and 7.5% being obese with BMI of 30+.

**Table 1:** Basic characteristics of the study population (*N*=59,503)

**Characteristic**	**N (%)**
Age group (yrs)	
Median (min - max)	44.2 (36.1 – 53.2)
15 – <25	3,862 (6.5)
25 – <35	9,710 (16.3)
35 – <45	16,734 (28.1)
45 – <55	16,516 (27.8)
55+	12,681 (21.3)
Sex	
Female	41,304 (69.4)
Male	18,199 (30.6)
District	
Handeni	6,603 (11.1)
Kilindi	2,282 (3.8)
Korogwe	9,776 (16.4)
Lushoto	6,035 (10.1)
Mkinga	2,723 (4.6)
Muheza	11,444 (19.3)
Pangani	3,319 (5.6)
Tanga	17,321 (29.1)
Facility Level	
Hospital	8,659 (18.2)
Health Center	28,293 (59.4)
Dispensary	10,687 (22.4)
BMI, kg/m^2^	
<18.5	2,686 (4.5)
18.5 – <25	45,307 (76)
25–<30	7,076 (12)
30+	4,434 (7.5)
WHO stage	
I	12,120 (24)
II	7,730 (15.2)
III	25,217 (49.5)
IV	5,889 (11.6)
CD4 count, cells/mm^3^	
<350	8,082 (28)
350 – 500	6,143 (22)
500+	14,102 (50)
Marital status	
Cohabiting	924 (1.7)
Divorced	9,564 (17.4)
Married	28,602 (52)
Single	15,972 (29)
ART duration (yrs)	
<=1	2,375 (4.0)
>1	57,128 (96.0)
Adherence	
Good	57,480 (96.6)
Poor	2,023 (3.4)
Regimen	
First line	58,176 (98.0)
Second line	1,256 (2.0)
DTG/TLD based drug	
Yes	54,564 (91.7)
No	4,939 (8.3)
VLR suppression failure	
No	57,213 (96.0)
Yes	2,290 (4.0)

At the time of the study, more than 61% of the study participants were in the WHO HIV stage III and IV and 24% were in WHO stage I. Meanwhile, seventy two percent had >350 CD4 count, cells/µL.

RETRACTED

Fifty-two percent (28,602) of the study participants were married, 29% single, 17.4% divorced and 1.7% cohabiting.

Of these adult clients, 96% were found to be on ART medication for more than one year and only 4% (2,375) on ART in less than a year but more than six (6) months. Furthermore, 96.6% of clients were well adhering to the ART drugs.

Based on regimen used, 98% were using first line ART drugs and only 2% were on second line ART. Ninety eighty percent (58,176) were initiated on Dolutegravir (DTG) based regimen mainly being Tenofovir, Lamivudine and Dolutegravir (TLD) about 91.7% while the rest were non based DTG regimen.

Ninety six percent (57,213) of the study participants were found be virally suppressed i.e having plasma viral load <1,000cp/ml and 4% not virally suppressed. That means, having higher plasma viral load level >1,000 cp/ml.

Table 2, shows a summary of risk factors/determinants associated with plasma virologic failure among adult clients on ART at Tanga region. In the multivariate model, the youngest group (15 - <25 years) were found to have 2.8 times risk of virologic failure which is statistically significant (HR: 2.82, 95% CI 1.96 – 4.04, *P* value < 0.0001) as compared to other groups with >35 years. The analysis shows significant risk of Virologic failure decrease with increasing age.

**Table 2:** Risk factors for viral load suppression failure among patients on ART in Tanga

Characteristics	Univariate HR 95% CI	*P* Value	Multivariate HR 95% CI	*P* value
Age group (yrs)				
15 – <25	2.40 (2.10 – 2.77)	<0.0001	2.82 (1.96 – 4.04)	<.0001
25 – <35	Reference		Reference	
35 – <45	0.84 (0.74– 0.95)	0.009	0.81 (0.60 – 1.10)	0.29
45 – <55	0.64 (0.56 – 0.73)	<0.0001	0.58 (0.43 – 0.79)	<0.0001
55+	0.53 (0.45 – 0.61)	<0.0001	0.41 (0.28 – 0.57)	<0.0001
Sex				
Female	Reference		Reference	
Male	1.13 (1.03 – 1.23)	0.008	1.00 (0.82 – 1.22)	0.97
BMI group, kg/m^2^				
<18.5	2.25 (1.95 – 2.60)	<.0001	1.69 (1.23 – 2.30)	<0.0001
18.5 – <25	Reference		Reference	
25 - <30	0.73 (0.63 – 0.85)	<.0001	0.65 (0.48 – 0.88)	
30+	0.51 (0.41 – 0.63)	<.0001	0.37 (0.23 – 0.59)	
WHO stage				
I	Reference		Reference	
II	1.34 (1.15 – 1.57)	0.885	1.43 (1.00 – 2.04)	0.15
III	1.28 (1.13 – 1.45)	0.233	1.07 (0.78 – 1.46)	0.03
IV	1.84 (1.58 – 2.16)	<.0001	1.60 (1.12 – 2.24)	0.008
CD4 count, cells/mm^3^				
<350	3.31 (2.87 – 3.82)	<0.0001	2.61 (2.12 – 3.23)	<.0001
350 – 500	1.51 (1.26 – 1.80)	0.02	1.76 (1.39 – 2.26)	0.40
500+	Reference		Reference	
Marital status				
Cohabiting	0.88 (0.65 – 1.20)	<0.13	1.04 (0.56 – 1.95)	0.488
Divorced	0.59 (0.54 – 0.65)	<0.0001	0.70 (0.57 – 0.87)	0.02
Married	Reference		Reference	
Single	0.57 (0.50 – 0.66)	<0.0001	0.84 (0.64 – 1.11)	0.66
District				
Handeni	1.05 (0.91 – 1.21)	0.578	1.39 (1.02 – 1.91)	0.02
Kilindi	2.11 (1.78 – 2.49)	<0.0001	1.66 (1.15 – 2.40)	0.006
Korogwe	0.95 (0.84 – 1.08)	0.193	0.88 (0.66 – 1.15)	0.07
Lushoto	0.91 (0.78 – 1.06)	0.08	0.81 (0.56 – 1.17)	0.06
Mkinga	0.76 (0.61 – 0.96)	0.004	0.75 (0.46 – 1.14)	0.06
Muheza	0.75 (0.66 – 0.86)	<0.0001	0.99 (0.61 – 1.62)	0.75
Pangani	1.05 (0.87 – 1.26)	0.73	1.35 (0.88 – 2.06)	0.17
Tanga	Reference		Reference	
Facility Level				
Hospital	Referenc		Reference	
Health Center	1.02 (0.89 – 1.15)	0.39	1.02 (0.78 – 1.33)	0.56
Dispensary	1.11 (0.96 – 1.29)	0.08	1.20 (0.86 – 1.67)	0.23
ART duration (yrs)				
<=1	1.33 (1.11 – 1.61)	0.0027	1.14 (0.79 – 1.65)	0.47
>1	Reference		Reference	
Adherence				
Good	Reference		Reference	
Poor		<0.0001	1.98 (1.80 – 2.18)	<0.0001
DTG/TLD				
Yes	Reference		Reference	
No	9.34 (8.54 - 10.2)	<0.0001	11.8 (9.74 – 14.3)	<0.0001
Regimen				
First line	Reference		Reference	
Second line	4.33 (3.67 – 5.11)	<0.0001	0.61 (0.44 – 0.85)	0.003

In the univariate model; Male clients were found to have statistically significant with 13% increased risk of virologic failure (HR: 1.13, 95% CI 1.03 – 1.23, *P* <0.008 as compared to female clients. Meanwhile, clients who were found to be underweight (BMI<18.5) had increased risk 1.69 times as compared to clients whom were found to have BMI >18.5. Normal weight or above were found to be protective against virologic failure.

RETRACTED

Clients with WHO stage III and IV had significant risk of virologic failure (HR: 1.25, 1.60, 95% CI 0.78 – 1.46; 1.12 – 2.24; *P* value 0.03, 0.008) respectively as compare to clients on WHO stage I and II. Additionally, clients whom were found to have CD_4_ count <350 cells/mm^3^ had 2.61 times risk of developing virologic failure (HR: 2.61, 95% CI 2.12 – 3.23; *P* value <0.0001) as compared to clients with CD_4_ > 350+ cells/mm^3^. Having more CD_4_ cells/mm^3^ were found to be protective against Virologic failure.

On marital status variable, being divorced were found to be significantly protective by 30% against the risk of virologic failure as compared to other marital status (RR: 0.70, 95% CI 0.57 – 0.87, *P* < 0.02.

Meanwhile, adult clients from Kilindi and Handeni Districts were found to be at risk significantly of having virologic failure as compared to other districts (HR: 1.66, 95% CI 1.15 – 2.40, *P* = <0.006; HR:1.39, 95% CI 1.02 – 1.91) due to nomadic nature of the clients.

RETRACTED

Poor ART adherence has 1.98 times risk to develop virologic failure as compared to client who had good adherence (HR: 1.98, 95% CI 1.80 – 2.18, *P* < 0.0001).

Not being on DTG based regimen was found to increase the risk of virologic failure 11.8 times as compared to using DTG regimen (HR: 11.8, 95% CI 9.74 – 14.3, *P* < 0.0001) while using second line regimen was found to be significantly protective by 39% against the risk of virologic failure (HR: 0.61, 95% CI 0.44 – 0.85, *P* = 0.003).

## Discussion

This study aim to describe determinants of virologicalfailure among adults (>15 year and older) who are on ART and attending health facilities in Tanga region. We found that 96% of adult (>15 years) were virally suppressed (<1,000 copies/ml) as compared to 4% whom were not virally suppressed. Further analysis demonstrated determinants associated with virological failure that includes; age, gender, BMI, late WHO stage, CD4 count levels, marital status, ART duration of less than one year, poor drug adherence, DTG based drug and regimen (first line or second line).

Our multivariate model, show youngest group (15 - <25 years) were found to have 2.82 times risk of developing virologic failure which was statistically significant (HR: 2.82, 95% CI 1.96 – 4.04, *P* value < 0.0001) as compared to other age groups. The analysis shows significant risk of virologic failure decrease with increasing age. Behavioral factors such as missing clinic on scheduled dates, school attendance, self-stigma, alcoholism and missing medication were contributing factors [15]. A study conducted in South Africa, show similar results where only 68% of young adults were virally suppressed [1, 15, 16]. Another study from Mexican shows, clients >30 years were statistically significant associated with better viral suppression levels as compared to young age group [17]. Additionally, a study from Cambodia show statistically significant factors associated with virologic failure among young age group (15 – 17years) that included attending adult clinic where young adults feel uncomfortable asking questions regarding their HIV status and care; those whom are cared by caregivers and relatives had more risk of being unsuppressed as compared to those taken care by parents; lack of enough understanding of HIV care and treatment; forgetfulness to take medication timely and self-stigma [15, 16, 18–21].

On marital status; divorced clients were statistically significant at reduced risk of virologic failure by 30% as compared to those who are cohabiting and single (HR: 0.70, 95% CI 0.57 – 0.87, *P* = 0.02). A study from China show a significant association among married and divorced with less likelihood of having virologic failure [18]. Additional studies also show marriage and divorced are associated with viral load suppression. Marriage tend to ensure stable environment for treatment support from a partner [16, 18, 19].

RETRACTED

Clients with WHO stage IV had significant risk of virologic failure (HR: 1.60, 95% CI 1.12 – 2.24, *P* value = 0.008) as compare to clients on WHO stage I, II and III. A study done in Malaysia, shows advanced WHO HIV stage IV was associated with high advance AIDS disease and opportunistic infections leading to increased comorbidities. Advanced HIV diseases are associated with risk of virologic failure and opportunistic infections with poor immunologic and virologic outcomes in HIV patients [22]. Meanwhile, WHO advanced stage shows hazard risk 1.8 times as compared to early HIV WHO stages [23].

Furthermore, clients with CD4 <350 cell/mm^3^ were at more risk (2.61 times) to develop virologic failure as compared to clients with CD4 >350 cell/mm^3^. A Switzerland study shows having CD4 >350 cell/mm^3^ were more protective by 50% with less virologic failure [23]. Meanwhile, adult clients 40+ years were found to have higher CD_4_; with female having higher CD_4_ levels as compared to male clients [22].

Being poorly adherent to the ARV regimen had 1.98 times increased risk of viral suppression failure (Hazard Risk: 1.98, 95% CI 1.80 – 2.18), *P* < 0.0001 which was statistically significant. Studies, show good adherence of >95% to ARV is directly proportional to Viral Load suppression and in return help to reduce progression of HIV/AIDS disease. Poor drug adherence was associated with poor prognosis, higher rate of morbidity and mortality [24, 25]. Moreover, a study from Switzerland shows clients with missing at least a dose was mostly associated with frequent missing as compared to those who never missed a dose [23]. It was found that, good ART adherence was associated with good social economic status and more evident in elderly clients >40+. And adherence was much better with clients using single tablet regimen as compared to multi tablet regimen [26, 27].

Our analysis shows, clients not being on DTG based regimen were found to increase the risk of virologic failure by 11.8 times as compared to those using DTG regimen (HR: 11.8, 95% CI 9.74 – 14.3, *P* < 0.0001) while using second line regimen was found to be significantly protective by 39% against the risk of viral load suppression failure (HR: 0.61, 95% CI 0.44 – 0.85, *P* = 0.003). Several studiesshow effectiveness of DTG based regimen in having shorter time to viral suppression. DTG based regimens were found to be superior to non DTG based therapy in reducing viral load to suppression levels and better tolerated by clients especially with single combination tablet therapy [28–33].

RETRACTED

Meanwhile, clients from Kilindi and Handeni Districts are at significant higher risk of having virologic failure as compared to other districts 39% and 66% respectively. Other studies, have found highly mobile communities such as pastoralist, fishermen and refugees were found to have lower viral suppression associated with treatment failure and/or interruption of treatment [27, 34, 35].

## Limitation of the study

Firstly, these findings rely mainly on secondary data obtained from CTC2 database. Patient information were extracted from files documented in the database which may subject to errors and incomplete documentation. These may underestimate the true proportional of clients who are truly suppressed. Second, since its secondary data; we are unable to distinguish the confounders which may affect the determinants of viral suppression.

Lastly, adherence was not measured by pill count method to identify exact number of pills taken or untaken.

## Conclusion

Our study revealed several variables which were found to be statistically significant associated with viral load suppression failure such as age, advanced WHO stage, CD4 count levels, ART adherence as well as DTG regimen. Intense measures are needed to be advocated and implemented to reach the marginalized population such as younger age group 15-24 years who are sexually active to help mitigate the spread of HIV and protect their future.

Several studies have found DTG based regimen to be superior to non DTG based therapy in reducing viral load to acceptable suppression levels within short time and better tolerated by clients [36, 37]. We therefore, advocate the active use, affordability, accessibility of DTG based regimen in reducing viral load to acceptable suppression levels within short time which are as well better tolerated by clients especially with single combination tablet therapy.

## Abbreviations

AIDS: Acquired Immunodeficiency syndrome
ART: Antiretroviral Treatment
BMI: Body Mass Index
CTC: Care and Treatment Center
DTG: Dolutegravir
HIV: Human Immunodeficiency Virus
LTFU: Lost to Follow up
NACP: National AIDS Control Program
PLHIV: People Living with HIV
RNA: Ribonucleic Acid
TACAIDS: Tanzania Commission for AIDS
THIS: Tanzania HIV Impact Survey
TLD: Tenofovir, Lamivudine and Dolutegravir
UNAIDS: United Nation for AIDS
VLS: Viral Load suppression
WHO: World Health Organization
